The article "The Effect of Copaiba Oil Odor on Anxiety Relief in Adults under Mental Workload: A Randomized Controlled Trial" was published in 2022. Journal: Evid Based Complement Alternat Med.

# The Effect of Copaiba Oil Odor on Anxiety Relief in Adults under Mental Workload: A Randomized Controlled Trial

**DOI:** 10.1155/2022/3874745

**Published:** 2022-03-20

**Authors:** Nan Zhang, Jie Chen, Wenyan Dong, Lei Yao

**Affiliations:** ^1^School of Design, Shanghai Jiao Tong University, 800 Dong Chuan Rd., Shanghai, China; ^2^Aromatic Plant R&D Center, Shanghai Jiao Tong University, 800 Dong Chuan Rd., Shanghai, China; ^3^dōTERRA (Shanghai) Commercial Co., Ltd, 699 West Nanjing Rd., Shanghai, China

## Abstract

**Background:**

Aromatherapy has been proved to be effective in alleviating anxiety in practices and research. Recently, copaiba oil (CPO) is popular in the market and is recommended for anxiety relief in aromatherapy practice. However, relevant scientific research is still lacking.

**Methods:**

A randomized controlled trial was designed to evaluate the anxiety-relieving effect of CPO inhalation in 22 adults. Jojoba oil was used as the control treatment. N-back and mental arithmetic tasks were used as stress stimulation. CPO or control intervention was carried out after the n-back training phase. The State-Trait Anxiety Inventory (STAI), EEG activities, physiological indexes including heart rate (HR), blood pressure (BP), blood oxygen saturation, and salivary cortisol were assessed in different phases of the experimental process.

**Results:**

There was no significant difference in the change of HR and BP between the CPO and control groups before odor intervention. The S-AI scores of the CPO treated participants decreased after the n-back and mental arithmetic tests and were significantly lower than those of the participants who received control treatments. The HR and salivary cortisol of participants who received CPO intervention significantly decreased during the n-back and mental arithmetic tests. Furthermore, a remarkable decrease of beta wave activity was observed in the left midfrontal region (F3) when the participant received the CPO intervention.

**Conclusion:**

The study's findings supported that the CPO odor showed beneficial effects on alleviating anxiety based on several indicators in subjective, physiological, and EEG measurements.

## 1. Introduction

Essential oils are derived from aromatic plants and are composed of various volatile chemical components. In aromatherapy, odor molecules enter the nasal cavity and attach to specific olfactory receptors on olfactory neurons. Such combination generates action potentials, initiates signal transduction, and further affects the neural activities in the limbic system that are closely related to anxiety and depression regulation [1]. In addition, essential oil compounds can easily enter the blood circulation by inhalation or massage application because of their small molecular weights and strong permeability.

In aromatherapy practices, the use of some essential oils could quickly relieve anxiety, stress, or other negative emotions [2]. At present, many studies provided evidence for the anti-anxiety effects of essential oils from citrus fruit peels [3], lavender [4], rose [5], and so on through either animal tests or clinical trials. In the history of the aromatherapy practice, resinous essential oils are also considered to be beneficial to the nervous system. However, there is little research on the emotion regulation effect of resin essential oils. Frankincense extracts have been proved to be anxiolytic in a previous preclinical test [6].

Copaiba balsam is the resin of the *Copaidera* genus, which is common in the Amazon region. Copaiba oil (CPO) is extracted from its resin by hydrodistillation. The content of *β*-caryophyllene could reach more than 50% in the CPO [7]. Because of its anti-inflammatory [8], skin-healing-promoting effect [9], and anti-parasitic properties [10], CPO has been widely used in folk medicine. The relevant pharmacological properties have been confirmed by modern scientific research in recent years. For example, CPO (3%) cream application could effectively prevent mechanical tenderness induced by UVB radiation in mice [7]. When given the CPO to volunteers suffering from hand arthritis by massage, the time of subjects completing dexterity tasks was significantly reduced, and the pain score decreased by approximately 50% compared to the control treatment [11].

*β*-Caryophyllene, which is the main component of CPO, has been proved to be anxiolytic in many previous studies [12]. It was thought to be a CB2 receptor, potent-selective agonist. Therefore, it could be speculated that CPO might have the function of anxiety-relieving. A recent animal study showed that intraperitoneal administration of CPO had an acute anxiolytic effect [13]. However, there is no evidence suggesting that the inhalation of the CPO has an anti-anxiety effect.

Cortisol produced in the adrenal cortex is the main glucocorticoid in the human body. It is released by the hypothalamic-pituitary-adrenal axis in response to various psychological stimuli. Many research had proved that essential oils with anxiolytic effects could attenuate the plasma corticosterone in animals [14] and decrease the salivary cortisol in clinical trials [15, 16]. Electroencephalogram (EEG) has a more direct relationship with brain activity. It has been used to study the relationship between olfactory stimulation and emotion. Several EEG studies have demonstrated significant alterations in activities of alpha waves (7.5–12.5 Hz) or beta waves (12.5–30 Hz) after the intervention of essential oils [17, 18]. In addition, heart rate (HR) and blood pressure (BP) are often considered to be related to anxiety. In many clinical studies of essential oils, these two indicators were positively correlated with anxiety [19, 20].

Therefore, the aim of this study was to investigate the efficacy of CPO inhalation for anxiety-relieving in a clinical trial. N-back and mental arithmetic tasks were carried out as mental workload and stress stimulation. The State-Trait Anxiety Inventory (STAI) was used as a self-report of anxiety. EEG, salivary cortisol, as well as several physiological indexes were recorded during the experiment.

## 2. Materials and Methods

### 2.1. Participants and Randomization

A randomized controlled trial was designed to evaluate the anxiety-relieving effect of inhalation of CPO. Jojoba oil, an almost odorless oil, was used as the control treatment. The study was approved by the Research and Ethics Offices of the Shanghai Jiao Tong University (No. H2021148I).

The study was conducted on the campus of Shanghai Jiao Tong University. Subjects were recruited through social-oriented electronic questionnaires. Subjects were eligible if they were aged 18–40 years old, with no nasal diseases, no medical conditions that could affect the sense of smell, no history of allergy to essential oils, and no history of taking psychotropic drugs in recent three months. Furthermore, female subjects should not be in the stage of preparation for pregnancy or pregnancy to avoid any potential affection by the odors. The informed consent forms were signed by the 22 eligible participants. The subjects (5 men and 17 women) were randomly assigned to the CPO group (*n* = 11) and the control group (*n* = 11). Practitioner and participant blinding were not considered possible, due to the nature of the odor intervention. The participants were not informed of when the odor was released in the experiment.

### 2.2. Materials and Intervention

CPO was provided by the doTERRA (Shanghai) Commercial Co. Ltd. Jojoba oil was provided by the Aromatic Plant R&D Center of Shanghai Jiao Tong University. An incense diffuser that could directly atomize pure essential oil and control the release time was used.

A separate space (1.7 × 1.7 × 1.85 m) was used as the test space. A chair and a small table were placed in this test space. The subject could finish the questions on a computer screen placed on the table. The incense diffuser was placed on the ground of the corner so that subjects would not notice it easily. When entering the aromatherapy intervention progress, the experimenter will start the incense diffuser and atomize the copaiba oil into the air. The working mode of the incense diffuser was set at every 60 s followed by a pause for 5 sec.

### 2.3. N-Back and Mental Arithmetic Tasks

*The n-back task.* N-back test is a kind of mental load task [21], in which subjects are asked to monitor a series of briefly presented stimuli and decide in each trial if the currently presented stimuli were the same as those presented one or more trials before [22]. In this study, a 300-s 1-back task was used as stress stimulation. All participants performed the 1-back task two times, for the first time as a training session, and the second time as a test session. The n-back task field was a square separated into smaller squares with lines (3 × 3 squares) shown on the computer screen. During the task, a visual stimulus accompanied with an auditory stimulus (a single letter) was randomly presented 500 ms in one of the squares every 3 s. The subjects should find a match of the position and color of the current image and the letter sound in the auditory to those shown one step earlier. The task was held through an online website (https://brainscale.net/dual-n-back). The participants were prompted on the computer screen if they choose a wrong answer.

#### 2.3.1. Mental Arithmetic Task

The participants were required to finish a 5 min mental arithmetic task containing 30 trials of 3-digit addition on the computer screen. Each trial lasts 10 s. The task was held through an online website (https://brainscale.net/mental-math). The participants would be prompted on the computer screen if they filled in a wrong answer.

### 2.4. Measurements of Physiological Index and Saliva Cortisol

HR, systolic blood pressure (SBP), and diastolic blood pressure (DBP) were measured by a digital blood pressure monitor (Omron). Blood oxygen saturation (SpO_2_) was measured by a finger clip oxygen saturation tester (Heal Force).

The saliva of the subjects was collected by EP tube and centrifuged at 8,000 rpm, 4°C for 10 min. The supernatant was collected and stored at −80°C. A human cortisol Elisa kit (Elabscience, China) was used to evaluate the cortisol content in the saliva. All operations were carried out strictly according to the instructions of the kit.

### 2.5. EEG Recording and Spectrum Analysis

The EEG was recorded using the eego™ mylab system (eego miniEE-401, ANT Neuro, Inc.). A cap (waveguard) was positioned on the subject using the standard 10–20 system. The electrode gel was applied onto electrode sites that were located at midfrontal (F3 and F4), central (C3 and C4), Fpz, Cz, and Pz. FCz was used as the reference electrode. Impedances were brought below 10K ohms. EEG signals were acquired at a sampling rate of 500 Hz. EEG data were digitally filtered offline to a 1–30 Hz bandwidth. The EEG data were edited for artifact using software asalab 4.10.2. Separate EEG relative power of alpha and beta spectral bands in the midfrontal and central brain regions were analyzed. Alpha and beta wave activities were highly related to anxiety mood change [17, 23]. Previous studies reported that brain activity in the prefrontal cortex was strongly linked to anxiety [24], and excessive power at beta frequencies around electrode sites C3, CZ, and/or C4 could be observed when both anxiety and problems with attention occurred [25]. Therefore, the relative power of each of the alpha (7.5–12.5 Hz) and beta (12.5–30 Hz) spectral bands was expressed as a percentage (%) of the total spectral power within the 1–30 Hz window, as previously reported [26].

### 2.6. Self-Report Measures

The STAI was compiled by Charles D. Spielberger et al. The first edition was published in 1970 and translated into Chinese in 1988. The scale is a self-assessment scale, which consists of 40 descriptive questions and is divided into 2 subscales: (1) state anxiety scale (S-AI), including questions 1–20, which describes a usually transient unpleasant emotional experience, such as tension, fear, anxiety, and neuroticism, accompanied by hyperfunction of the nervous system and (2) trait anxiety scale (T-AI), including questions 21–40. Trait anxiety describes a relatively stable anxiety tendency as a personality trait with individual differences [27]. In this study, the STAI was used to measure the anxiety state of the participant.

A Likert scale ranging from −5 to 5 was used to self-evaluate the comfort of the environment odor in the test zoom at the end of the experimental procedure. A score of “5” to “−5” was assigned to the feeling of “very comfortable” to “very uncomfortable.” A five-level scale was used to self-evaluate the intensity of the environment odor. Scores of 1–5, respectively, represent “no smell,” “almost unrecognizable smell,” “slightly identifiable smell,” “easily identifiable smell,” and “strong smell.”

### 2.7. Experimental Procedure

The subjects were asked to avoid alcohol, nicotine, coffee, drugs, and any essential oil on the test day. Food intake was not allowed 1.5 h before the test. At the beginning of the test, subjects were asked to sit in a comfortable position. The EEG cap was positioned on the subject's head. After an adaptive sitting for 10 min, the subjects completed the baseline physiological parameters measurements including HR, BP, and blood oxygen saturation. Saliva was also collected. The EEG of the subject was recorded for 5 min with eyes closed.

The experimental procedure (Figure 1) was conducted in the following order. (1) The subjects were first given a 5 min training session of the n-back (*n* = 1) task. After training, the relevant physiological parameters were measured; saliva was collected; and the STAI scale was filled out. (2) Then, the EEG was recorded for 10 min with the subject's eyes closed. After 5 min, the odor of the essential oil or the jojoba oil was released into the space through an incense diffuser without informing the subject. The odor was released for a total of 20 min with a 5 s stop between every 60 sec. (3) Subjects then performed a 5 min n-back (*n* = 1) test and a 5 min rapid mental arithmetic task. The test results were given to the subjects after each task. Then, the EEG of the subject was recorded for 5 min with eyes closed. The relevant physiological parameters of subjects were measured again. Saliva was also collected. The STAI scale and environmental odor evaluation were filled out. All the work tasks and STAI scales were performed on a computer.

### 2.8. Identification of Constituents of the Copaiba Oil

The copaiba oil was diluted 10 times with a solution of ethanol and n-hexane (1:1, v/v). Gas chromatography/mass spectrometer (GC/MS, Agilent 7890B-5977 A) was used to analyze the constituents of copaiba oil. The GC was filled with a methylpolysiloxane nonpolar column (DB-WAX: 30 m × 0.25 mm × 0.25 *μ*m). The GC conditions were as follows: carrier gas, helium (1 mL/min); split rate, 10:1; and column temperature, 50°C for 3 min, 50°C to 120°C at 4°C/min, then 120°C for 10 min, 120°C to 220°C at 2°C/min, then 220°C for 12 min. The MS conditions were as follows: inlet line temperature, 280°C; source temperature, 230°C; and mass spectra electron impact, 70 eV. Individual components were identified from the mass spectral library (NIST14).

### 2.9. Statistical Analysis

Statistical analyses were conducted using SPSS 14.0 software. Unpaired two-tailed Student's *t*-test was used when comparing data of subjects in different groups. Paired two-tailed Student's *t*-test was used when comparing data collected at different times of the same subject. Statistical significance was defined if *p* value <0.05.

## 3. Results

### 3.1. Chemical Composition of the Copaiba Oil

Terpenes were the main ingredients of the CPO (Table 1). The CPO contained 55.93% caryophyllene, 10.41% *α*-copaene, 6.81% trans-*α*-bergamotene, and 5.46% humulene. The sum of the relative contents of the compounds (relative content above 1%) was 93.03%.

### 3.2. The STAI Score Change after the CPO Intervention

The results of STAI showed that the CPO odor environment could well alleviate the anxiety of participants compared to the control odor environment under the same stress task stimulation (Table 2). The STAI, S-AI, and T-AI scores of the two groups showed no statistically significant difference after the n-back training (*p* > 0.05). Overall, compared with the n-back training session, the tension of participants in each group in the n-back and mental arithmetic test session showed a decreased trend. The S-AI score of the CPO group was significantly lower than the control group (*p* < 0.05). The STAI, S-AI, and T-AI scores of the CPO group significantly decreased after the mental arithmetic test (*p* < 0.05). Only the T-AI score decreased significantly after the mental arithmetic test in the control group (*p* < 0.05).

Pre- and posttests mean the time point after n-back training and after the mental arithmetic test, respectively. The value represents means ± SEM. Paired two-tailed Student's *t*-test was used for the comparison between pre- and posttest. Unpaired two-tailed Student's *t*-test was used for the comparison between the control and CPO group. ^*∗*^*p* < 0.05 compared with the score of the participant before the task test. ^#^*p* < 0.05 compared with the score of the control group in the same experiment step.

### 3.3. The Physiological Change after the CPO Intervention

CPO odor had no statistically significant effect on participants' BP (Table 3). However, it could significantly affect the HR of the participant. During the n-back and mental arithmetic test sessions, the HR of the CPO group decreased, and the change was significant compared to the control group (*p* < 0.05). SpO_2_ levels of the CPO group showed an upward trend during the n-back and mental arithmetic sessions (Table 3).

The salivary cortisol level of the CPO group significantly decreased from 374.0 ng/ml to 130.4 ng/ml (*p* < 0.05) during the n-back and mental arithmetic test sessions. On the contrary, salivary cortisol of the control group showed an upward trend (Figure 2). The salivary cortisol level of the CPO group was significantly lower than those of the control group (*p* < 0.05). These results indicated that CPO odor relieved the stress of participants during the test session.

The calculation method of the changes of SBP, DBP, HR, and SpO_2_ is: the change (%) = (post – pre)/pre × 100%. The value represents means ± SEM. Training: n-back training session. Test: n-back and mental arithmetic tasks test session.

### 3.4. Effects of CPO Intervention on EEG Power Spectrum Pattern

The EEG data of four 5-min stages of the experiment were analyzed (Figures 3 and 4). There was a significant decrease of beta (12.5–30 Hz) power (*p* < 0.05) in the F3 region of the CPO group during the first 5-min odor intervention stage compared with the posttraining stage (after the n-back training and before the odor intervention; Figure 3(c)). A decreased trend of beta (12.5–30 Hz) power could also be observed in the F4 region during the CPO intervention but showed no significant difference compared with it in the posttraining stage (*p* > 0.05). These changes were not observed in the control treatment group who received odorless jojoba oil treatments (Figures 3(a)–3(d)). In the first 5-min odor intervention stage, the alpha (7.5–12.5 Hz) power in F3, F4, C3, and C4 regions showed a trend of decrease, but there was no statistical significance (Figures 3(a) and 3(b) and Figures 4(a) and 4(b)). There were no significant changes of beta (12.5–30 Hz) power (*p* > 0.05) in C3 and C4 regions during each task stage (Figures 4(c) and 4(d)).

### 3.5. Evaluation of the Perception of the Environmental Odor

The two groups of participants showed differences in the perception of odors in the environment. The score of odor comfort of the CPO group was higher than that of the control group, but there was no significant difference (*p* > 0.05). In terms of the odor intensity, the participants could clearly sense a stronger aroma of the CPO. The intensity score of the CPO group was significantly higher (*p* < 0.05) than that of the control group (Figure 5).

## 4. Discussion

In this study, n-back and mental arithmetic tasks were used as stress stimulations, and the effect of CPO odors on anxiety-relieving was evaluated. The participants first experienced the training phase of the n-back task and then received a continuous test phase of the n-back and mental arithmetic task. Before and after these two stages, the psychological and physiological indexes of the participants were collected.

The CPO odor showed some significant effects on alleviating anxiety that were shown in several indexes in subjective, physiological, and EEG measurements. The STAI scale had been used in several previous studies to evaluate the effect of essential oil interventions on anxiety relief. Acute inhalation of essential oils with floral, fruity, or herb smell, such as pelargonium [28], bergamot [29], and salvia [30] oils, was proved to help reduce the STAI score. In the present study, the STAI score of the control and CPO group showed no difference after the n-back training. The STAI score of the CPO group significantly decreased after the mental arithmetic test, while the control group did not have the change. These results indicated that the woody odor of CPO might help relieve the anxiety of the participants compared to an odorless treatment. S-AI and T-AI, which are two subscales of STAI, represent state anxiety and trait anxiety, respectively [31]. The S-AI score only decreased after the mental arithmetic test in the CPO group. Moreover, the S-AI score of the CPO group was significantly lower than that of the control group. These results indicated that the CPO odors can alleviate the state anxiety of the participants during the experiment.

The changes in HR and BP are related to people's tension. The sympathetic response of the autonomous system leads to an increase in BP and HR. In some research, these physiological markers had negative relationships with blood oxygen saturation [32]. Some previous studies have reported that smelling or massaging essential oils such as ylang-ylang, bitter orange, and lavender could reduce HR [33], and a pleasant smell could bring a decrease in HR [34]. The BP change was observed after a few essential oil interventions such as ylang-ylang and bitter orange oil that were thought to be sedative [19, 20]. There was no significant difference in the change of HR, BP (both diastolic and systolic blood pressure), and blood oxygen saturation between the two groups before and after the n-back training stage without odor intervention. After the odor intervention, the HR changes of participants in the CPO group were significantly different from those in the control group during the n-back and mental arithmetic task stage. The HR of the control group showed an upward trend in the test stage, while that of the CPO group showed a downward trend. These results showed that the inhalation of CPO could alleviate participants' tension. Many essential oils containing *β*-caryophyllene, such as *Baccharis uncinella* and *Ocimum basilicum* oils showed some sedative effects [35]. The decrease of HR might be related to the inhalation of this ingredient in the oil. The CPO odor did not affect the BP and blood oxygen saturation of the participants. This was similar to a previous study that rosemary and lavender oil could help relieve anxiety and reduce radial pulse but did not reduce the BP of participants during a math test [36]. In another study, significant changes in BP were observed in the lavender oil group postoperatively [37]. This inconsistency of results might be due to different experimental tasks design.

Cortisol is a salivary endocrinological stress marker [16]. The hypothalamic-pituitary-adrenal axis (HPA) is one of the main components of the stress system. Activation of hypothalamic-pituitary-adrenal axis is associated with the secretion of cortisol [38]. Saliva collection is much more convenient than blood collection, so it has been used in many clinical studies. Several previous studies showed that some essential oils could affect the cortisol contents in saliva [15, 39]. In the present study, the content of salivary cortisol of the control group increased in the n-back and mental arithmetic test stage, while the salivary cortisol of the CPO group decreased. The salivary cortisol of the CPO group was also significantly lower than that of the control group. These results were consistent with the data presented in HR and STAI self-report, which indicated that the CPO intervention could alleviate the anxiety of the participants.

In general, the beta wave activity decreases during the drowsiness state and increases with a high alertness level [40]. Many studies have demonstrated that essential oils affect the EEG spectrum power in rats and humans. In a previous study, inhalation of essential oil of chamomile, which was thought to be anxiolytic, led to a decrease of frontal beta wave activities in females [41]. In the present study, a remarkable decrease of beta wave power was observed in the left midfrontal region (F3) when the participant received the CPO intervention. These results indicated that inhalation of CPO odor could help relax and relieve anxiety, which was consistent with the results of STAI, HR, and cortisol. A decreased trend of alpha wave power was shown in the F3, F4, C3, and C4 regions of the CPO group after receiving the odor intervention. These results were consistent with a previous study in which the subjects who received rosemary intervention and obtained lower anxiety scores exhibited decreasing alpha and beta power [18].

However, this study has potential limitations. In one of our unpublished studies on odor preference, there was no significant gender difference in the preference of CPO. However, the sample size of the present study was small, and there were more females than males. Whether there were gender differences in the anxiety-relieving function of CPO could not be discussed in this study. Furthermore, in the process of odor intervention, the essential oil molecules in the experimental environment space were accumulated due to the continuous running of the aroma diffuser. The odor concentration was not strictly controlled. This problem is common in many clinical studies of aromatherapy [42]. A large sample size and an environment with controlled odor concentration will be helpful to explore if the anxiolytic functions vary at different concentrations in further study.

## 5. Conclusion

CPO with a woody odor is popular in aromatherapy these years and is recommended for anxiety-relieving in aromatherapy practice. In the present study, a randomized controlled trial was designed to evaluate the anxiety-relieving effect of CPO inhalation in 22 adults. N-back and mental arithmetic tasks were used as stress stimulation. The results showed that the CPO odor could well alleviate the anxiety of participants compared to the control environment. The S-AI score of the CPO treated group decreased after the n-back and mental arithmetic test, and it was significantly lower than that of the control group. The HR and salivary cortisol of participants who received CPO intervention significantly decreased during the n-back and mental arithmetic tests. Furthermore, a remarkable decrease of beta wave activity was observed in the left midfrontal region (F3) when the participant received the CPO intervention. Studies using a larger sample size and environments with controllable odor concentrations will be helpful to further explore the anxiolytic function of CPO.

## Figures and Tables

**Figure 1:** The experimental procedure.

**Figure 2:** The change of salivary cortisol in control and CPO groups during three sessions of the experiment. s1: before the training of the n-back task; s2: after the training of the n-back task; and s3: after the n-back and mental arithmetic task. Values represent the mean ± SEM. ^*∗*^*p* < 0.05, paired two-tailed Student's *t*-test was used. ^#^*p* < 0.05, unpaired two-tailed Student's *t*-test was used.

**Figure 3:** The frontal alpha (7.5–12.5 Hz) and beta (12.5–30 Hz) activities (% of total 1–30 Hz spectrum power) in F3 (a) and (c) and F4 (b) and (d) during four 5-min stages of the experiment. Pretraining: before the n-back training task; posttraining: after the n-back training task; intervention: immediately after receiving CPO or control treatment; and posttask: after the mental arithmetic test task. Values represent the mean ± SEM. ^*∗*^*p* < 0.05. Paired two-tailed Student's *t*-test was used.

**Figure 4:** The frontal alpha (7.5–12.5 Hz) and beta (12.5–30 Hz) activities (% of total 1–30 Hz spectrum power) in C3 (a) and (c) and C4 (b) and (d) during four 5-min stages of the experiment. Pretraining: before the n-back training task; posttraining: after the n-back training task; intervention: immediately after receiving CPO or control treatment; and posttask: after the mental arithmetic test task. Values represent the mean ± SEM. Paired two-tailed Student's *t*-test was used.

**Figure 5:** The subjective evaluation of the comfort and intensity of the odors. The median line of the histogram represents the average of the value. ^*∗*^*p* < 0.05. Unpaired two-tailed Student's *t*-test was used.

**Table 1:** Main chemical compounds of the CPO and its released odor in the air.

Retention time	Compound	Relative content (%)
20.07	Caryophyllene	55.93
16.83	*α*-Copaene	10.41
19.83	trans-*α*-Bergamotene	6.81
22.27	Humulene	5.46
23.81	Germacrene D	4.38
26.06	*δ*-Cadinene	2.01
24.82	*β*-Bisabolene	1.98
15.78	*α*-Cubebene	1.84
21.34	*γ*-Elemene	1.55
16.15	*γ*-Muurolene	1.34
23.07	*δ*-Elemene	1.32
Sum		93.03

The table only lists the compounds with a relative content above 1%.

**Table 2:** The STAI score change after CPO or control treatment.

	Control group (*n* = 11)		CPO group (*n* = 11)	
	Pretest	Posttest	Pretest	Posttest
STAI score	87.1 ± 5.8	82.8 ± 5.9	78.7 ± 4.0	72.9 ± 3.6^*∗*^
S-AI score	37.9 ± 3.2	36.5 ± 3.7	33.5 ± 1.8	32.3 ± 1.6^*∗*#^
T-AI score	49.2 ± 3.2	46.3 ± 3.1^*∗*^	45.2 ± 3.0	40.6 ± 3.1^*∗*^

**Table 3:** Comparison of the change of four physiological indexes between control and CPO group in n-back training and n-back test sessions.

		Training session	Test session
SBP change (%)	Control group (*n* = 11)	1.23 ± 1.64	−0.71 ± 1.21
	CPO group (*n* = 11)	4.55 ± 1.28	−1.31 ± 1.83
	*p* value	*0.13*	*0.79*

DBP change (%)	Control group (*n* = 11)	3.51 ± 2.84	−0.60 ± 2.23
	CPO group (*n* = 11)	4.06 ± 2.46	−1.12 ± 1.52
	*p* value	*0.88*	*0.85*

HR change (%)	Control group (*n* = 11)	−3.64 ± 2.56	3.52 ± 2.82
	CPO group (*n* = 11)	3.54 ± 4.89	−4.15 ± 2.97
	*p* value	*0.21*	*0.04*

SpO_2_ change (%)	Control group (*n* = 11)	0.1 ± 0.29	−0.18 ± 0.51
	CPO group (*n* = 11)	−0.36 ± 0.60	1.05 ± 0.47
	*p* value	*0.49*	*0.09*

The calculation method of the changes of SBP, DBP, HR, and SpO_2_ is: the change (%) = (post – pre)/pre × 100%. The value represents means ± SEM. Training: n-back training session. Test: n-back and mental arithmetic tasks test session.

## Data Availability

Data generated or analyzed during this study are included in this article. Further enquiries are available on reasonable request to the corresponding author.

## Additional Points

*Highlights.* (i) A randomized controlled trial indicated that inhalation of copaiba oil could help relieve the anxiety of the participant during mental workload. (ii) The STAI scores and physiological indexes related to anxiety including heart rate and salivary cortisol decreased after the participant received the copaiba oil inhalation treatment. (iii) A decrease in left midfrontal beta wave activities of EEG was observed during the copaiba oil treatment.
